The article "Efficacy of Novavit in ameliorating the neurotoxicity of propionic acid" was published in 2020. Journal: Transl Neurosci.

# Efficacy of Novavit in ameliorating the neurotoxicity of propionic acid

**DOI:** 10.1515/tnsci-2020-0103

**Published:** 2020-05-26

**Authors:** Sarah I. Bukhari, Hanan Alfawaz, Abeer Al-Dbass, Ramesa Shafi Bhat, Nadine MS Moubayed, Wadha Bukhari, Sohair A. Hassan, Nada Merghani, Samar Elsamaligy, Afaf El-Ansary

**Affiliations:** Department of Pharmaceutics, College of Pharmacy, King Saud University, Riyadh, Saudi Arabia; Department of Food Science and Nutrition, College of Food Science and Agriculture, King Saud University, Riyadh, Saudi Arabia; Department of Biochemistry, College of Science, King Saud University, Riyadh, Saudi Arabia; Department of Botany and Microbiology, College of Science, King Saud University, Riyadh, Saudi Arabia; Central Laboratory, Female Center for Medical Studies and Scientific Section, King Saud University, P O Box 22452, Riyadh, Saudi Arabia; Therapeutic Department, National Research Centre, Dokki, Egypt; Department of Pharamaceutics and Industrial Pharmacy, Helwan University, Ain Helwan, Cairo, Egypt

**Keywords:** autism, fatty acids, oxidative stress, gut microbiota, Novavit.

## Abstract

Oxidative stress, abnormal fatty acid metabolism, and impaired gut microbiota play a serious role in the pathology of autism. The use of dietary supplements to improve the core symptoms of autism is a common therapeutic strategy. The present study analyzed the effects of oral supplementation with Novavit, a multi-ingredient supplement, on ameliorating oxidative stress and impaired lipid metabolism in a propionic acid (PPA)-induced rodent model of autism. Male western albino rats were divided into three groups. The first group is the control, the second group was given an oral neurotoxic dose of PPA (250 mg/kg body weight/day) for 3 days and then received buffered saline until the end of the experiment. The third group received Novavit (70 mg/kg body weight/day for 30 days after the 3-day PPA treatment). Markers of oxidative stress and impaired fatty acid metabolism were measured in brain homogenates obtained from each group. Novavit modulation of the gut microbiota was also evaluated. While PPA induced significant increases in lipid peroxides and 5-lipoxygenase, together with significantly decreased glutathione, and cyclooxygenase 2, oral supplementation with Novavit ameliorated PPA-induced oxidative stress and impaired fatty acid metabolism. Our results showed that the presence of multivitamins, coenzyme Q10, minerals, and colostrum, the major components of Novavit, protects against PPA-induced neurotoxicity.

## 1 Introduction

Autism is a neurodevelopmental disorder characterized by abnormal social interactions with sensory dysfunction and repetitive and stereotyped behaviors. Prevalence estimates are 1–2 diagnoses per 100 individuals. Nutritional interventions for autism treatment aim to stimulate social interaction and other autistic phenotypic features. These may be managed by caregivers and professionals, with parents often functioning as cotherapists [1].

The article "Efficacy of Novavit in ameliorating the neurotoxicity of propionic acid" was published in 2020. Journal: Transl Neurosci.

Several biomarker studies have reported significant abnormalities in antioxidant status and fatty acid metabolism in autistic children [2,3,4,5]. Autistic patients from Saudi Arabia have much lower levels of glutathione (GSH) and polyunsaturated fatty acid and elevated lipid peroxides, saturated fatty acids, prostaglandins, and 8-isoprostane compared to the age-matched controls [6,7]. A previous study showed that children with autism from Egypt had lower plasma levels of polyunsaturated fatty acids, except linoleic acid, compared to the healthy controls [8].

Prostaglandins, leukotrienes, and thromboxanes are metabolites produced by cyclooxygenases (COXs) and 5-lipoxygenase (ALOX5) that mediate the inflammatory response [9,10]. Each of these lipid mediators influence neural development, aging, and neurodegeneration [11].

Cytoplasmic phospholipase A2 alpha (cPLA2α) is an enzyme that hydrolyzes phospholipids to mobilize arachidonic acid (AA) for eicosanoid production, a major class of neuroinflammatory signaling molecules. In addition, cPLA2α also regulates the composition of membrane phospholipids to allow for proper membrane structure and function [12]. An important contributor to membrane structure and function is a phosphatidylinositol (PI) species which contains AA at both the sn-1 and sn-2 positions [13]. In addition to an important role in innate immune function, PI may also act as a short-lived acceptor for incorporation of AA into various cellular phospholipid classes [14]. Owing to the high AA content, PI is also a major source for AA release via cPLA2α in activated immune cells [13,14,15,16]. The importance of phospholipids in normal brain function suggests that membrane lipid replacement may be an effective treatment strategy to repair phospholipids in membranes of organelles, cells, and organs [17].

Animal models are typically used to evaluate pathological mechanisms of disease and to suggest possible treatment strategies that target affected metabolic pathways. Although autism is a human disorder, rodent models can contribute to the understanding of the etiology of autism and to evaluate therapeutic agents [18]. Previous studies [7,19] proposed that brain infusion or oral administration of propionic acid (PPA) to rat pups could induce many of the biochemical characteristics observed in individuals with autism. Moreover, histopathological changes, such as neuronal loss, hyaline bodies, and astrogliosis, together with several behavioral traits such as hyperactivity, impaired social interaction, reduced exploratory activity, and increased repetitive behaviors, have been recorded [19,20,21].

The article "Efficacy of Novavit in ameliorating the neurotoxicity of propionic acid" was published in 2020. Journal: Transl Neurosci.

It is well accepted that the composition of microbiota regulates the levels of short-chain fatty acids (SCFAs), including acetic acid, PPA, and valeric acid. Wang et al. [22] reported that the levels of these SCFAs and ammonia in stool were considerably higher in children with autism when compared with healthy controls. Additionally, Shaw [23] reported higher concentrations of urinary 3-(3-hydroxyphenyl)-3-hydroxypropaonic acid in children with autism spectrum disorder (ASD) compared with controls. Song et al. [24] suggested that the source of this compound might be multiple species of anaerobic bacteria of the *Clostridium* genus. Recently, the involvement of microbiota in ASD pathogenesis and the possibility to use as a target to treat this disorder were greatly encouraged [25]. This information supports the use of PPA for induction of autism in a rodent model.

As autism etiology is multifactorial and the disorder is characterized by complex pathophysiology, the use of complex supplements might be successful as a treatment strategy. Vitamin B6 is widely used to decrease behavioral problems observed in autism [26], but the mechanism is not fully understood. Vitamin B6 plays a critical role in the synthesis of many neurotransmitters, such as gamma aminobutyric acid, serotonin, dopamine, and noradrenalin, and vitamin B6 supplementation can enhance many neurotransmitter systems affected in autism [27,28].

Ali et al. [29] produced a developmental vitamin D (DVD)-deficiency model of autism. This DVD-deficiency model may prove relevant for investigation of possible therapeutic strategies to reverse the abnormality of direct regulation of the fetal/placental immune response during pregnancy and improve impaired steroid biosynthesis, which are two accepted mechanisms relating DVD to autistic phenotypes. Although DVD may only represent one environmental contributor to autism, the ability to intervene safely and effectively during pregnancy might help to avoid the development of autistic phenotypes.

Similar results were observed with respect to vitamins E, C, and A and folic acid. Multiple studies correlated micronutrient deficiencies with development of autism [3,30]. Adams et al. [31] recommended vitamin/mineral supplementation as a valuable nutritional intervention strategy for children with autism. Supplementation resulted in remarkable improvements in GSH levels, oxidative stress, sulfation, methylation, ATP, NADH, and NADPH.

The article "Efficacy of Novavit in ameliorating the neurotoxicity of propionic acid" was published in 2020. Journal: Transl Neurosci.

Coenzyme Q10 (CoQ10), a lipid-soluble benzoquinone, exerts intracellular antioxidant activity that preserves membrane phospholipids and mitochondrial proteins from free radical-induced oxidative damage [32]. CoQ10 supports mitochondrial functions such as electron transport, which is critical for ATP production [33]. Previous studies have shown that autistic children with CoQ10-restricted diet either due to sensory sensitivities or due to therapeutic measures suffer from mitochondrial dysfunction [34,35,36] and that CoQ10 supplementation in mice is usually accompanied by remarkable improvement in behavior [37]. Our most recent work showed that insufficient serum CoQ10 might play a role in autism pathophysiology [38].

Novavit is a nutritional supplement that acts as an antiaging and detoxification agent. This unique cellular food component contains a large quantity of embryonic predifferentiated duck stem cells as well as several minerals and vitamins to support health. Furthermore, Novavit contains many amino acids such as arginine, proline, lysine, carnitine, cysteine, and inositol. In addition, it contains CoQ10, folic acid, and a variety of essential vitamins such as vitamins B, E, D, and C that function with amino acids to enhance collagen synthesis and improve scar healing. Table 1 demonstrates the ingredients of Novavit (https://www.novavitcomplexusa.com/).

**Table 1:** Ingredients of Novavit complex

	Compound
Vitamins	Vitamin A Vitamin D Cholecalciferol (D3) Vitamin E Vitamin C
	Water-soluble vitamins:
	Vitamin C. Ascorbic acid Vitamin B1. Thiamine Vitamin B2. Riboflavin Vitamin B3. Niacinamide. Nicotinic acid. Vitamin PP Vitamin B5. Pantothenic acid. Vitamin W Vitamin B6. Pyridoxine. Vitamin B8. Biotin Vitamin B9. Folic acid Vitamin B12. Cyanocobalamin
	Glutathione Oligoelements such as beta-carotene, folic acid, biotin and lysine, proline, carnitine, arginine, Cysteine, CoQ10, alpha lipoic acid, French marine pine extract, bioflavonoids, and colostrum
Minerals	The natural clay’s basic chemical structure is MgO·Al_2_O_3_·5SiO_2_·*n*H_2_O with high content of magnesium, silica, potassium, calcium, phosphates, iron oxide, aluminum, manganese, and titanium. This clay has special benefits such as detoxifying action, remineralizing action, and is extremely absorbent
Other	Embryonic predifferentiated duck stem cells

In addition to the discussion of neurological effects and disorders related to PPA and food supplement deficiency, it is important to highlight the critical role that the gut microbiota play in human metabolism and health [39]. Intestinal bacterial composition is important in digestion, protection against invading pathogens, and regulating immunity and metabolism of host cells [39]. Any disturbance in this composition can lead to the development of diseases and may trigger an autoimmune response. Diet also has an impact on the gut microbial composition, mainly noted on the following day [40], where a high number of certain bacterial species will dominate and suppress other strains [41].

The article "Efficacy of Novavit in ameliorating the neurotoxicity of propionic acid" was published in 2020. Journal: Transl Neurosci.

We hypothesized that the use of Novavit as a complex nutritional supplement could minimize oxidative stress and neuroinflammation induced by PPA by modulating antioxidant defense. In addition, Novavit suppressed the growth of the *Clostridia* species, thus altering the impaired gut microbiota. We analyzed lipid peroxidation and antioxidant markers in addition to PLA2, COX2, ALOX5, phospholipids, leukotrienes, and prostaglandins in brain homogenates of PPA-treated rats as a rodent model of autism and characterized the gut microbial composition alteration prior and following Novavit dosage.

## 2 Methods

### 2.1 Animals

Twenty-one young male western albino rats (80–120 g) were obtained from King Saud University Riyadh. Rats were randomly allocated to the following groups. Group I, the control group, was given phosphate-buffered saline (PBS). Group II was given oral buffered PPA (250 mg/kg body weight/day for 3 days) followed by PBS solution until the end of the study. Group III was given Novavit complex (70 mg/kg body weight/day for 30 days after the 3-day PPA treatment), a product of Novavit, Inc., USA [6]. All animals were reared in a controlled temperature environment and were given access to food and water under standard laboratory conditions.


**Ethical approval:** The research related to animal use has been complied with all the relevant national regulations and institutional policies for the care and use of animals. All protocols were approved by the ethics committee of King Saud University.

### 2.2 Sample collection

#### 2.2.1 Brain tissue

After sacrifice, the brain tissue was collected, washed, and homogenized with distilled water (1/10 by volume/weight ratio). After homogenization, the tissue was centrifuged at 3,500 rpm for 15 min. The clear supernatant obtained was used for the following assays.

### 2.3 Biochemical analyses

#### 2.3.1 Spectrophotometric analysis

- The method of Ruiz-Larrea et al. [42] was used for lipid oxidation, which is estimated by the formation of thiobarbituric acid reactive substances.
- The method of Jagota and Dani [43] was used for vitamin C analysis.
- The method of Beutler and Yeh [44] was used to assay GSH using 5,5′-dithiobis 2-nitrobenzoic acid with sulfhydryl compounds to produce a relatively stable yellow color.

The article "Efficacy of Novavit in ameliorating the neurotoxicity of propionic acid" was published in 2020. Journal: Transl Neurosci.

#### 2.3.2 ELISA

- Sandwich ELISA principle was used to estimate phospholipase A2 and COX2. Kits from LSBio (Lifespan BioScience, Inc., North America) were used with a detection range of 3.12–200 and 0.156–10 ng/mL, respectively.
- Competitive ELISAs were used for estimation of leukotriene B4 and prostaglandin E2 (PGE2). Kits were purchased from Cayman Chemical Company (Ann Arbor, MI, USA), with the assay range from 3.9–500 and 7.8–1,000 pg/mL, respectively.

### 2.4 Microbiological analyses

#### 2.4.1 Collection and preparation of fecal samples

Fecal samples were collected from all animal groups before and after treatment and were stored at −80°C. One gram of fecal matter was homogenized using a sonicator for 30 s in 10 mL of 0.1 M pH 7.2 PBS. The solutions were then centrifuged at 4,500 rpm for 3 min at 4°C. One milliliter of the fecal supernatant was then serially diluted in 9 mL of sterile PBS solution four times [45].

#### 2.4.2 Bacterial enumeration and culturing

Nutrient agar (Oxoid) plates, MacConkey plates, blood agar plates, and plates containing cycloserine–cefoxitin fructose agar (CCFA) medium selective for *Clostridia* were used to grow bacteria using 100 µL of each of the prepared dilutions for every group of animals. Anaerobic jars containing 5% CO_2_ at 37°C were used for CCFA medium selective for *Clostridia*, with a 3-day incubation period. All other culture media were incubated at 37°C under aerobic conditions for 18–24 h. The experiment was repeated twice. The average number of bacteria per plate was recorded. Gram staining and biochemical tests were used to identify the bacterial strains.

### 2.5 Statistical analysis

Results are expressed as mean ± SD. All statistical comparisons between the groups were performed using one-way analysis of variance (ANOVA) tests with Dunnett’s test for multiple comparisons. Adjusted *P* values were also calculated by the Bonferroni test. Significance was assigned at the level of *P* < 0.05. Receiver-operating characteristic (ROC) curve and area under the curve (AUC), the degrees of sensitivity and specificity, and the cutoff values were evaluated using Pearson’s correlations.

## 3 Results

Table 2 and Figure 1 show mean ± SD and the percentage change in the measured parameters in the three studied groups. The PPA treatment significantly increased lipid peroxides by 11.72%, and ALOX5 level by 100.62%, compared to the control. In contrast, PPA-treated rats expressed GSH and COX2 at much lower levels than control rats, showing 22.65% and 20.14% decreases, respectively. Ascorbic acid, leukotriene B4, and PGE2 levels did not change significantly with PPA treatment. Treatment with Novavit reversed PPA-induced changes in GSH, PLA2, ALOX5, and COX2, as summarized in Figure 1 and Table 2.

The article "Efficacy of Novavit in ameliorating the neurotoxicity of propionic acid" was published in 2020. Journal: Transl Neurosci.

**Table 2:** Mean ± SD of the measured parameters in the three studied groups

Parameter	Group	N	Min.	Max.	Mean ± SD	Percentage change	*P* value^a^	*P* value^b^	*P* value^c^
Lipid peroxides	Control	7	0.47	0.52	0.50 ± 0.02	100			0.001
	PPA	7	0.52	0.59	0.56 ± 0.02	11.72	0.001	0.001	
	PPA + Novavit	7	0.51	0.57	0.55 ± 0.02	9.5	0.001	0.002	
Ascorbic acid	Control	7	23.94	28.42	25.83 ± 1.40	100			0.126
	PPA	7	23	26	24.02 ± 1.08	−7.01%	0.081	0.136	
	PPA + Novavit	7	22.89	29.21	25.07 ± 2.08	−2.93%	0.58	1	
Glutathione	Control	7	88.88	97.92	93.15 ± 3.27	100			0.001
	PPA	7	65.7	75.7	72.06 ± 3.50	−22.60%	0.001	0.001	
	PPA + Novavit	7	93.23	101.93	96.61 ± 3.49	3.71%	0.132	0.138	
PLA_2_	Control	7	1160	2091.9	1,441.00 ± 317.85	100			0.102
	PPA	7	1106	2290.1	1,852.28 ± 393.77	28.54%	0.064	0.107	
	PPA + Novavit	7	1120.1	1891.3	1,677.42 ± 296.25	16.41%	0.342	0.623	
ALOX5	Control	7	226.55	365.09	293.88 ± 46.28	100			0.001
	PPA	7	406.68	795.32	589.59 ± 126.69	100.62	0.001	0.001	
	PPA + Novavit	7	192.51	271.27	225.08 ± 27.98	−23.41%	0.21	0.369	
COX2	Control	7	73.98	92.33	81.66 ± 6.50	100			0.011
	PPA	7	54.96	72.6	65.21 ± 5.24	−20.14%	0.006	0.01	
	PPA + Novavit	7	60.42	95.63	75.55 ± 13.39	−7.48%	0.368	0.677	
Phospholipid (mM/g)	Control	7	13.08	21.62	16.76 ± 2.80	100			0.01
	PPA	7	7.35	16.13	12.21 ± 3.17	−27.14%	0.008	0.013	
	PPA + Novavit	7	11.75	15.77	13.10 ± 1.52	−21.82%	0.031	0.05	
Leukotriene B4 (pg/g)	Control	7	386.04	413.65	404.55 ± 9.39	100			0.001
	PPA	7	380.18	416.17	391.82 ± 12.40	−3.15%	0.239	0.424	
	PPA + Novavit	7	329.89	393.74	366.63 ± 21.83	−9.37%	0.001	0.001	
PGE2 (pg/g)	Control	7	238.99	381.8	267.42 ± 51.26	100			0.511
	PPA	7	239.91	253.47	244.75 ± 4.45	−8.48	0.443	0.833	
	PPA + Novavit	7	213.57	332.73	249.45 ± 40.75	−6.72	0.587	1	

^a^ *P* value between each group and the control group using Dunnett’s test as multiple comparisons.

^b^ *P* value between each group and the control group using Bonferroni test as multiple comparisons.

^c^ *P* value between all groups using one-way ANOVA.

**Figure 1:** Percentage change of all parameters in all groups compared to control.

Table 3 summarizes the Pearson’s correlation coefficients between the measured variables. Lipid peroxides negatively correlated with GSH expression (*P* < 0.003) and positively correlated with ALOX5 (*P* < 0.049). GSH negatively correlated with ALOX5 (*P* < 0.001) and positively correlated with COX2 (*P* < 0.001). ALOX5 negatively correlated with COX2 (*P* < 0.029).

**Table 3:** Correlations between the measured variables

Parameters	*R* (Person correlation)	Sig.	Significance
Lipid peroxides with glutathione	−0.442**	0.003	N^b^
Lipid peroxides with PLA_2_	0.554**	0.001	P^a^
Lipid peroxides with ALOX5	0.306*	0.049	P^a^
Ascorbic acid with phospholipid assay (mM/g brain tissue)	0.457**	0.002	P^a^
Glutathione with PLA_2_	−0.476**	0.001	N^b^
Glutathione with ALOX5	−0.804**	0.001	N^b^
Glutathione with COX2	0.488**	0.001	P^a^
PLA_2_ with ALOX5	0.345*	0.025	P^a^
ALOX5 with COX2	−0.338*	0.029	N^b^

^*^Correlation is significant at the 0.05 level.

^**^Correlation is significant at the 0.01 level.

^a^Positive correlation.

^b^Negative correlation.

The article "Efficacy of Novavit in ameliorating the neurotoxicity of propionic acid" was published in 2020. Journal: Transl Neurosci.

Table 4 presents the cutoff values, AUC, sensitivity, and specificity of each of the measured markers for the PPA-treated group and the PPA-treated group supplemented with Novavit. Most of the measured variables showed reasonable AUCs, specificity, and sensitivity as a marker of PPA neurotoxicity and/or the therapeutic effect of Novavit.

**Table 4:** ROC analysis of all variables in all groups

Parameter	Group	Area under the curve	Cutoff value	Sensitivity (%)	Specificity (%)	*p* value
Lipid peroxides	PPA	0.990	0.515	100.0	85.7	0.002
	PPA + Novavit	0.959	0.515	85.7	85.7	0.004
Ascorbic acid	PPA	0.837	24.865	85.7	85.7	0.035
	PPA + Novavit	0.673	24.605	57.1	85.7	0.277
Glutathione	PPA	1.000	82.290	100.0	100.0	0.002
	PPA + Novavit	0.796	93.192	100.0	71.4	0.064
PLA2	PPA	0.755	1527.55	85.7	85.7	0.110
	PPA + Novavit	0.735	1507.70	85.7	85.7	0.142
ALOX5	PPA	1.000	385.89	100.0	100.0	0.002
	PPA + Novavit	0.918	275.305	100.0	71.4	0.009
COX2	PPA	1.000	73.29	100.0	100.0	0.002
	PPA + Novavit	0.633	71.58	57.1	100.0	0.406
Phospholipid assay (mM/g brain tissue)	PPA	0.878	15.56	85.7	71.4	0.018
	PPA + Novavit	0.878	15.10	85.7	71.4	0.018
Leukotriene B4 (pg/g brain tissue)	PPA	0.796	397.435	85.7	85.7	0.064
	PPA + Novavit	0.959	396.854	100.0	85.7	0.004
PGE2 (pg/g brain tissue)	PPA	0.684	244.765	71.4	71.4	0.250
	PPA + Novavit	0.673	243.030	57.1	85.7	0.277

Fecal bacterial analysis from each of the animal groups in the study was performed and tabulated as an average of the bacterial count per plate. Data were compared between the groups before and after treatment with Novavit following PPA administration.

### 3.1 Microbial data

The microbial profile of all groups (Table 5 and Figures 2, 3) mainly consisted of *Staphylococcus aureus*, identified as a bacterium with a grape-like structure when observed under a microscope following gram staining. Very few enteric bacteria (gram-negative rod) were found during the study period following PPA and Novavit administration. Moreover, Novavit intake greatly decreased *Clostridium* sp.

**Table 5:** (a) Estimating colony count/plate after 3 days of PPA dose followed by Novavit intake. Day 0 following treatment with Novavit. (b) Estimated colony count/plate following PPA treatment (1 week). (c) Estimated colony count/plate at 3 weeks

(a)				
Isolated organisms	Media and incubation conditions	Novavit	PPA	Control (pretreatment)
*Staphylococcus* and/or bacilli (gram-positive cocci/rod and or gram-negative rod)	N.A./aerobic: 37°C/24 h	20	180	300
*Enterobacteriaceae* (gram-negative rod, lactose fermenters)	Mac/aerobic: 37°C/24 h	4	23	0
Gram-positive/gram-negative rod and cocci	Blood agar/aerobic: 37°C/24 h	4	120	100
*Clostridium* sp.	CCFA/anaerobic 37°C with 5% CO_2_	0	0	0

(b)			
Isolated organisms	Media and incubation conditions	Novavit	PPA
*Staphylococcus* and/or bacilli (gram-positive cocci/rod or gram-negative rod)	N.A./aerobic: 37°C/24 h	0	30
*Enterobacteriacea* (gram-negative rod, lactose fermenters)	Mac./aerobic: 37°C/24 h	0	3
Gram-positive/gram-negative rod and cocci	Blood agar/aerobic: 37°C/24 h	0	16
*Clostridium* sp.	CCFA/anaerobic 37°C with 5% CO_2_	0	0

(c)			
Isolated organisms	Media and incubation conditions	Novavit	PPA
*Staphylococcus aureus* (gram-positive cocci grape-like structure)	N.A/aerobic: 37°C/24 h	>300	20
*Enterobacteriaceae* (gram-negative rod lactose fermenters)	Mac./aerobic: 37°C/24 h	0	1
Gram-positive cocci or bacilli	Blood agar/aerobic: 37°C/24 h	200	10
*Clostridium* sp.	CCFA/anaerobic 37°C with 5% CO_2_	0	0

The article "Efficacy of Novavit in ameliorating the neurotoxicity of propionic acid" was published in 2020. Journal: Transl Neurosci.

**Figure 2:** Average bacterial plate count following PPA treatment (3 days).

**Figure 3:** Bacterial plate count (1 week of treatment).

## 4 Discussion

Nutritional deficiencies may play a chief role in autism because many patients are selective eaters with high sensitivity toward many foods, which might lead to inadequate intake of nutrients [46]. Thus, nutritional interventions can significantly help these patients [47,48,49]. Adams [50] reported that vitamins, minerals, amino acids, and specialty supplements are key components in the biomedical approach for the treatment of autism. The use of complex supplements could be beneficial in treating this disorder.

The results summarized in Table 2 demonstrate significant irregularities in biomarkers of oxidative stress following PPA administration. While Novavit was ineffective in reducing lipid peroxides, it potently increased vitamin C levels. Additionally, Novavit ameliorated decreased GSH levels in PPA-treated rats (*P* < 0.001) to levels not significantly different from the control group (*P* < 0.580). The recorded increase in GSH and vitamin C in Novavit-treated rats is likely due to vitamins B, C, D, and E contained in Novavit. Vitamin D is effective in increasing GSH levels in the brain through calcitriol upregulation of γ-glutamyl transpeptidase, the rate-limiting enzyme in GSH synthesis [51,52,53]. A recent review by Jia et al. [54] reported improvement in GSH levels in autistic patients treated with vitamin D. Moreover, the remarkable increase in GSH levels in Novavit-treated rat brains can be attributed to CoQ10 treatment (30 or 60 mg CoQ10/day for 100 days), an important component of the electron transport chain known to reduce GSH peroxidase enzymatic activity and improve gastrointestinal (GI) problems and sleep disorders in children with autism [55].

The article "Efficacy of Novavit in ameliorating the neurotoxicity of propionic acid" was published in 2020. Journal: Transl Neurosci.

Both glycine and glutamic acid, components of the tripeptide GSH, are readily available in the diet of most individuals. In contrast, cysteine is not readily available, making it the rate-limiting amino acid for GSH intracellular synthesis. In free amino acid form, cysteine is toxic and is broken down in the GI tract and the blood. Colostrum, the first milk secretion, is rich in cystine, a stable form of cysteine that can cross the blood–brain barrier (BBB). Based on this, colostrum is a unique component of Novavit that can explain the significant increases in GSH in Novavit-treated rats [56].

The brain is highly susceptible to lipid peroxidation due to the abundance of polyunsaturated fatty acids, high aerobic metabolism, and low levels of antioxidant enzymes [57]. Lipid peroxidation in the brain following administration of PPA may be responsible for PPA-induced neurotoxic effects [58]. Activation of phospholipase A2 as a phospholipid-hydrolyzing enzyme can contribute to depletion of brain phospholipids, potentially contributing to PPA-induced neurotoxicity [58]. Data summarized in Table 1 and Figure 1 demonstrate the activation of PLA2 with concomitant depletion of brain phospholipids in the PPA-treated groups. Moreover, Novavit reduced PLA2 activity, resulting in phospholipid replenishment.

The unexpected decreases in COX-2 and PGE2 in the PPA-treated rats (*P* < 0.005) (Table 2 and Figure 1) may be related to alteration in the gut microbiota (Table 5 and Figures 2, 3). COX2 plays a critical role in the adaptive cytoprotection response in GI mucosal cells. When the GI tract is inflamed in response to toxins resulting from pathogenic bacterial overgrowth, large amounts of prostaglandins (PGs) are produced at the sites of injury by rapidly induced COX2. This process typically aids in the healing process of the injured gut. Under these conditions, inhibition of COX2 should be avoided in patients who are vulnerable to GI inflammation (e.g., autistic patients) [59]. Moreover, enhanced BBB leakage also correlates with impaired markers of brain inflammation [60]. Animal models of autism support increased BBB permeability as a characteristic feature related to glutamate excitotoxicity as an etiological mechanism [61]. BBB disruption can affect influx and efflux of proteins and ions. This may contribute to the unexpected decrease in PLA2 and PGs in brains of PPA-treated animals [62,63]. This hypothesis agrees with the previous work of Qasem et al. [64,65] in which PLA2 and PG were markedly higher in the plasma of autistic patients compared to the controls. Novavit treatment increased COX2 to levels similar to the controls.

The article "Efficacy of Novavit in ameliorating the neurotoxicity of propionic acid" was published in 2020. Journal: Transl Neurosci.

Data summarized in Table 2 and Figure 1 demonstrate that in spite of a twofold increase in ALOX5 in PPA-treated rat pups, leukotriene B4 levels did not significantly change. Leukotriene B4 is an enzymatic hydration product of AA that can be conjugated and excreted. Novavit was effective in counteracting the effects of PPA as a neurotoxic mediator through a significant decrease in ALOX5 to levels comparable to controls. Leukotriene B4 was significantly lower in the Novavit-treated group compared to the controls.

Table 2 shows the Pearson’s correlations between the measured parameters. Positive correlations were found among PLA_2_, ALOX5, and lipid peroxides, with a concomitant negative correlation with GSH. These results confirmed the contribution of oxidative stress, impaired lipid metabolism, and neuroinflammation as neurotoxic mechanisms of PPA to the rodent model of autism and the therapeutic efficacy of Novavit as a multisupplement.

Table 4 summarizes the AUCs for all measured markers of PPA neurotoxicity and Novavit therapeutic potency. With few exceptions, most of the measured variables showed high AUCs with satisfactory specificity and sensitivity, which supports their use as valid markers.

Similarly, Novavit intake had a remarkable effect on the gut bacterial composition. Our study demonstrated that following the administration of Novavit, a mixture of vitamins B, E C, and D, and folic acid, the gut bacterial composition and the total bacterial count were altered with abundance of gram-positive bacteria (mainly *S. aureus*) on day 1, followed by an absence of bacterial growth (total bacterial number was (0) at week 1), then a subsequent reemergence of gram-positive bacteria. PPA administration resulted in increased bacteria number per plate on day 1 and throughout the experiment compared to Novavit-induced bacterial count, in agreement with the findings of Wu et al. [40]. However, both PPA and Novavit negatively impacted *Clostridium* sp., as this bacterium was absent in both treatment groups (Table 2 and Figures 2, 3).

Previous studies of germ-free and conventional rodents, and of human volunteers, reported that the gut microflora can synthesize vitamins such as vitamin K and vitamin B including biotin, pyridoxine, riboflavin, thiamine, cobalamin, folates, nicotinic acid, and pantothenic acid [66]. These vitamins are important for bacterial and mammalian metabolism. Magnúsdóttir et al. [67] explored the genomes of 256 common gut bacteria for the presence of eight vitamin B (including biotin, cobalamin, folate, pyridoxine, riboflavin, and thiamin) producers and found that each vitamin is produced by a different phylum, for instance, riboflavin was found to be mainly synthesized by the phylum Bacteroidetes, whereas Firmicutes had the ability to produce vitamin B. Previous studies of vitamin A and D deficiencies [68,69,70] revealed that some vitamins can interfere with the microbial gut composition and result in alteration of gut bacterial composition at the phyla levels in response to vitamin intake. Mandal et al. [70] noted that vitamin D intake increases the ratios of Actinobacteria/Proteobacteria, Proteobacteria/Firmicutes, whereas higher intake of vitamin E caused a decrease in the ratio of Proteobacteria/Actinobacteria and Firmicutes. At the genus level, Mandal et al. [70] observed that with fat-soluble vitamin intake, *Staphylococcus* was most abundant after vitamin E intake and lower with vitamin D intake, which agreed with the present data, where *Staphylococcus aureus* was the most abundant species encountered at the beginning and end of the experiments following Novavit. This is consistent with increased abundance of GSH as the main sulfur source for bacterial growth [71]. Furthermore, the presence of colostrum in Novavit, which is rich in antimicrobial peptides [72], is of nutritive importance, regulates GI disorders, and alters the gut microbiota, resulting in abundance of certain types of bacteria [73,74,75]. Interestingly, the presence of duck embryonic stem cells as a unique component of Novavit may increase its nutritional value and therapeutic efficacy. Because cell therapy is one of the most exciting fields in translational medicine, the effect of duck embryonic stem cells in Novavit can be related to its potency in downregulating certain proinflammatory cytokines, cytokine receptors, and cell cycle transcripts and upregulating signal transduction, cell adhesion, and cytoskeletal protein transcripts [76]. Moreover, under appropriate conducive conditions, populations of stem cells change to cells with features of neuronal-like tissues, which might explain the recorded potency of Novavit in the present study [76].

The article "Efficacy of Novavit in ameliorating the neurotoxicity of propionic acid" was published in 2020. Journal: Transl Neurosci.

The finding of the current study is of great support to our previous work in which vitamin D, CoQ10, vitamin B12, carnitine, and bioflavonoids (as major components of bee pollen) demonstrate significant potency in ameliorating PPA-induced persistent autistic features in the rodent model [77,78,79,80,81,82,83,84].

## 5 Conclusion

This study showed that Novavit, a multi-ingredient supplement usually given to modify risk factors associated with aging and disease, ameliorates PPA-induced neurotoxic in a rat model of autism. As only some products sold to consumers are validated scientifically, this study confirmed that multivitamins, CoQ10, minerals, and colostrum, components of Novavit, contribute to its potential use for the treatment of neurotoxicity and as prerequisite in translational medicine.

## 6 Limitations

There are two major limitations in this study that could be addressed in future research. First is the relatively small sample size, and second, the inability to measure the effectiveness of Novavit as a complex supplement in improving induced autistic behavior in the PPA-induced rodent model. Further studies using a larger number of subjects are required to determine whether the effect of substrate intake on gut microbiota is related to each substrate, nutrient alone, or food intake rich in these substrates.
